The article "Dapagliflozin Improves Diabetic Cardiomyopathy by Modulating the Akt/mTOR Signaling Pathway" was retracted in 2023. Reasons: unreliable results or conclusions; concerns about the data; concerns about the peer review; concerns about the citations.

# Dapagliflozin Improves Diabetic Cardiomyopathy by Modulating the Akt/mTOR Signaling Pathway

**DOI:** 10.1155/2022/9687345

**Published:** 2022-07-26

**Authors:** Mengxiang Ren, Dabin Pan, Dayong Zha, Zeyang Shan

**Affiliations:** ^1^Department of Cardiology, Yijishan Hospital, Wannan Medical College, Anhui Province, China 241001; ^2^Department of Cardiology, Wuhu Second People's Hospital, Anhui Province, China 241001; ^3^Department of Cardiology, Bengbu Second People's Hospital, Anhui Province, China 233000

## Abstract

**Background:**

Dapagliflozin can significantly improve heart failure, and Cx43 is one of the molecular mechanisms of heart failure. This study investigated the effect of dapagliflozin on Cx43 and Akt/mTOR signaling pathway in ventricular myocytes.

**Methods:**

A rat model of type 2 diabetes mellitus was established by high-fat diet combined with streptozotocin, and the animals were treated randomly with dapagliflozin. The morphological changes of the myocardium were observed by hematoxylin eosin staining, and the expression and distribution of Cx43 in ventricular myocytes were detected by immunohistochemistry. And Western blot determined the expressions of Cx43, Akt, mTOR, p62, and LC3 proteins in rat myocardium.

**Results:**

Compared with the normal control group, the heart rate of diabetic rats decreased significantly (*p* < 0.05), QRS wave of ECG widened, and QT interval prolonged (*p* < 0.05). Dapagliflozin treatment in diabetic rats resulted in improvements in these ECG indexes (*p* < 0.05) with early administration group obtaining greater efficacy than the late administration group (*p* < 0.05). In the normal control group, the cardiomyocytes were arranged orderly, and the expression of Cx43 was dense, uniform, and regular, which was higher than that in the intercalated disc. In the diabetic control model group, the cardiomyocytes were enlarged and presented disorderly with detection of Cx43 in the cytoplasm. Early use of dapagliflozin better improved these myocardial tissue lesions. Of note, as diabetic rats exhibited decreased expression of Cx43, Akt, and mTOR (*p* < 0.05), increased p62 expression (*p* < 0.05), and decreased LC3-II/I ratio (*p* < 0.05), administration of dapagliflozin partially reversed the expression of the above proteins (*p* < 0.05) with greater improvement in the early administration group compared with the late administration group (*p* < 0.05).

**Conclusions:**

Dapagliflozin increases the expression of Cx43 in cardiomyocytes of diabetic rats and thereby alleviates heart failure partly through regulating the Akt/mTOR signaling pathway.

## 1. Introduction

Dapagliflozin is a new oral hypoglycemic drug and an inhibitor of sodium-glucose cotransporter 2 (SGLT2) to reduce the reabsorption of glucose by the kidney and promote the excretion of glucose in urine by inhibiting SGLT2 in the kidney [1]. In recent years, studies have depicted its cardioprotective effect, apart from good hypoglycemic effect [2, 3].

The article "Dapagliflozin Improves Diabetic Cardiomyopathy by Modulating the Akt/mTOR Signaling Pathway" was retracted in 2023. Reasons: unreliable results or conclusions; concerns about the data; concerns about the peer review; concerns about the citations.

For patients with heart failure and a reduced ejection fraction (HFrEF), regardless of the presence or absence of diabetes, administration of dapagliflozin significantly decreases the risk of worsening heart failure or death from cardiovascular [4–6]. Without obvious side effects on these patients [6], dapagliflozin shortens hospitalization for heart failure in patients with and without HFrEF [7].

Gap junctions have a wide range of physiological functions and play a key role in excitatory and nonexcitatory tissues. Connexin (Cx) is one of the most important proteins of cardiac gap junction. Cx43 is the most important transmembrane aqueous channel connexin expressed in ventricular muscle as it forms an ion channel between cardiomyocytes and maintains the conduction of electrical signals between cardiomyocytes. Its normal expression and distribution are an important guarantee for normal electrical activity and coordination of cardiac diastolic and systolic functions [8].

Cx43 mRNA and protein are significantly downregulated in left ventricular in patients with end-stage heart failure caused by ischemic cardiomyopathy and idiopathic dilated cardiomyopathy. Congestive heart failure is associated with a significant decrease in the level of Cx43, the main gap junction protein in the left ventricle, which may lead to the enhancement of arrhythmia and systolic dysfunction [9].

Diabetic cardiomyopathy (DCM) is initially described as a human pathophysiological condition of heart failure without coronary heart disease, hypertension, and valvular heart disease. Of note, recent studies in animal models of diabetes have found that declined myocardial cell function is an important mediating mechanism for heart failure [10]. Changes in Cx43 content and distribution possibly contribute to alterations in cardiac function [11], while its expression in cardiomyocytes is closely related to the Akt/mTOR signaling pathway, an important pathway involved in oncogenesis and the cellular processes of metabolism [12]. Studies have found that dapagliflozin can affect autophagy through the Akt/mTOR signaling pathway [13, 14].

Low-after-high glucose promotes cardiomyocyte H9c2 cell autophagy through PI3K/Akt/mTOR and MEK/ERK1/2 signaling pathways, thereby downregulating Cx43. Chloroquine inhibited autophagy and reversed the downregulation of Cx43. U0126 inhibited ERK activation and decreased autophagy protein expression, but increased Cx43 expression, indicating that Cx43 expression is closely related to autophagy, and the mechanism is related to PI3K/Akt/mTOR and MEK/ERK1/2 signaling pathways [15]. As such, when the primary vascular smooth muscle cell (VSMC) is stimulated with ox-LDL, inhibiting Cx43 may activate VSMC autophagy to inhibit foam cell formation by inhibiting the PI3K/AKT/mTOR signaling pathway [16].

The article "Dapagliflozin Improves Diabetic Cardiomyopathy by Modulating the Akt/mTOR Signaling Pathway" was retracted in 2023. Reasons: unreliable results or conclusions; concerns about the data; concerns about the peer review; concerns about the citations.

Dapagliflozin can significantly improve cardiac function, but whether it has an effect on the expression of Cx43 in cardiomyocytes remains elusive. In this study, we investigated the effects of dapagliflozin on Cx43 expression and Cx43-related Akt/mTOR signaling pathway in cardiomyocytes of type 2 diabetic rats.

## 2. Methods and Materials

### 2.1. Materials

Specific pathogen-free (SPF) grade 4-week-old (70-80 g) male SD rats were purchased from Hunan Changsha Tianqin Biotechnology Co., Ltd. Common feed, high-fat feed, and streptozotocin (STZ) were all obtained from Beijing Boai Port Biotechnology Co., Ltd. Cx43 antibody (#AF0137), mTOR antibody (#AF6308), AKT antibody (#AF6261), GAPDH antibody (#T0004), *β*-actin antibody (#AF7018), LC3 antibody (#AF5402), p62 antibody (#AF5384), goat anti-rabbit IgG (#S0001), and goat anti-mouse IgG (#S0002) were all purchased from Affinity Biosciences (Affinity Biosciences Milwaukee, WI 53224, America). Dapagliflozin was provided by AstraZeneca Pharmaceutical Co., Ltd.

### 2.2. Animal Procedure and Drug Administration

The experimental procedure was reviewed and approved by the experimental animal welfare and ethics committee of Wannan Medical College (LLSC-2020-144). Rats were housed in the SPF-grade animal room of Wannan Medical College.

The animals were randomly divided into two groups: normal groups and model group. Type 2 diabetes mellitus (T2DM) model was established by feeding with high-fat diet first for 4 weeks and then one-time lower left abdominal intraperitoneal injection of 35 mg/kg STZ. One week later, a random blood glucose measurement > 16.7 mmol/L indicated successful establishment of diabetes models. The control group was fed a normal diet for 4 weeks and then received injection of the same amount of citric acid buffer.

The control group was randomly divided into normal control group (group A, *n* = 10) and normal administration group (group B, *n* = 10). The diabetic model group was randomly split into diabetic control group (group C, *n* = 10), early administration group (group D, *n* = 10), and late administration group (group E, *n* = 10). After modeling, group B and group D began administration with dapagliflozin 1 mg/kg/day via gavage, and the other groups were gavaged with the same amount of normal saline. After 8 weeks, group E began to receive dapagliflozin 1 mg/kg/day via gavage, when the treatment of the other groups remained unchanged until the end of the animal experiment.

The article "Dapagliflozin Improves Diabetic Cardiomyopathy by Modulating the Akt/mTOR Signaling Pathway" was retracted in 2023. Reasons: unreliable results or conclusions; concerns about the data; concerns about the peer review; concerns about the citations.

### 2.3. General Phenotypes and Electrocardiogram (ECG) Observation

During feeding, an electronic balance (Shanghai Minqiao Scientific Instrument Company, China) and blood glucose meter (ACCU-CHEK, Roche, USA) were used to monitor the weight and blood glucose of the rats in each group every week, and their mental state, diet, and urine output were observed and recorded. After 16 weeks, under anesthesia with sodium pentobarbital (Beyotime, China) at a dose of 40 mg/kg, after supine fixation of the limbs, a needle was inserted into the subcutaneous layer of the rats and connected to an RM6240E multichannel physiological signal acquisition and processing system (Chengdu Instrument Factory, China); the electrocardiogram (ECG) was recorded, and the heart rate, QRS wave width, and QT interval data of the rats in each group were measured three times with the average values taken.

### 2.4. Assay of NT-Pro-Brain Natriuretic Peptide (NT-proBNP, BNP)

After establishment of the diabetic model, the BNP content in the blood of all rats was determined in strict accordance with the instructions of the ELISA Kit (Shanghai Enzyme-Linked Biotechnology Co., Ltd). We set 6 standard wells and 2 blank wells, and the rest of the wells were used as sample wells to be tested. 50 *μ*L standard of 6 concentration gradients was added to the standard wells, 40 *μ*L diluents and 10 *μ*L plasma supernatant of rats in normal control group and diabetes model group to each sample well in sequence, and 50 *μ*L diluent to the blank wells. After that, the ELISA plate was shaken slowly, and 100 *μ*L of enzyme labeled reagent was added into the sample holes and standard holes rather than the blank hole. Then, after the ELISA plate was completely sealed with sealing film, it was incubated in the incubator at 37°C for 60 min. After incubation, the sealing film was torn off and the liquid in the hole was poured out. We added 300-200 *μ*L of washing solution and then poured it out three times and pat the liquid in the hole as dry as possible on the clean filter paper. Then, 50 *μ*L reagent A (H_2_O_2_) and 50 *μ*L reagent B (R&D, DY999) were added into each hole in turn. The ELISA plate was shaken slowly and then sealed with the plate sealing film, covered with tin foil paper, and placed in the incubator for 20 min. Then, 50 *μ*L of termination liquid was added into each hole. When the liquid changes from blue to yellow, this step should be completed quickly. We used the microplate reader to detect the OD value, which were zeroes according to the value of the blank hole, and measured the absorbance at the wavelength of 450 nm of each hole, that is, the OD value of each hole. The data were processed by ELISA Calc software, and the concentration of BNP in each hole was calculated according to the standard curve of the standard.

The article "Dapagliflozin Improves Diabetic Cardiomyopathy by Modulating the Akt/mTOR Signaling Pathway" was retracted in 2023. Reasons: unreliable results or conclusions; concerns about the data; concerns about the peer review; concerns about the citations.

### 2.5. Detection of Serum Lipid Levels

Blood sample was collected from the rat abdominal aorta and centrifuged at 4000 rpm for 10 minutes. The supernatant was transferred to a 2 mL EP tube and stored at -20°C. Plasma concentrations of total cholesterol (TC), triglycerides (TGs), low-density lipoprotein cholesterol (LDL-C), and high-density lipoprotein cholesterol (HDL-C) were detected by an automatic biochemical analyzer (Nanjing Ono Medical Equipment Co., Ltd., China).

### 2.6. Hematoxylin and Eosin (HE) Staining and Immunohistochemistry

After euthanasia, each rat's heart was removed and washed with normal saline, and the water was removed with filter paper. Partial ventricular muscle tissues were retained and fixed in EP tubes filled with paraformaldehyde for one week. These tissues were dehydrated, embedded in paraffin, sliced at a thickness of 5 *μ*m, dewaxed, dehydrated, and sealed. Morphological changes in the myocardium were observed with HE staining.

Dehydrated and dewaxed glass slides were sealed with 3% H_2_O_2_ at room temperature for 10 minutes and subjected to antigen retrieval. After rewarming, the slides were incubated with the primary antibodies (Cx43) 4°C overnight and then with the corresponding secondary antibodies for 30 minutes at room temperature. After the slides were incubated in streptavidin-biotin complex, the reaction was carried out at 37°C for 20 minutes. The slides were restained with hematoxylin, sealed with glycerol, and observed under a microscope.

### 2.7. Western Blot Analysis

The ventricular tissue (100 mg) was cut, and total protein samples were extracted from the tissues according to the instructions of the total protein extraction kit (Beyotime, China). With protein concentration detection, the proteins were separated by 8%, 10%, and 12% sodium dodecyl sulfate polyacrylamide gel electrophoresis and transferred to PVDF membranes (Beyotime, China). After being blocked for 2 hours with 5% skimmed milk powder, the membranes were washed and incubated in the primary antibody (Akt, mTOR, Cx43, LC3, and p62) working solution and shaken overnight at 4°C. After being washed, the membranes were probed with the corresponding secondary antibodies (GAPDH, *β*-Actin) at room temperature for 2 hours. According to the reagent instruction manual, the membranes were treated with a developer (Affinity, USA) and visualized on a Tanon-5500 cold CCD fluorescence image analysis system (Tanon, China). Each detection was repeated at least 3 times for protein quantification. The density of the signal was quantified with ImageJ (version 1.8.0).

The article "Dapagliflozin Improves Diabetic Cardiomyopathy by Modulating the Akt/mTOR Signaling Pathway" was retracted in 2023. Reasons: unreliable results or conclusions; concerns about the data; concerns about the peer review; concerns about the citations.

### 2.8. Statistical Analysis

SPSS 21.0 (SPSS, Inc., Chicago, IL, USA) was used for statistical analysis. The measurement data are expressed as the mean ± standard deviation (^−^*x* ± *s*). The means between multiple groups were compared by one-way analysis of variance (ANOVA), and the comparison between two groups was performed with the least significant difference (LSD) test. The inspection level was set at *α* = 0.05, and *p* < 0.05 indicated statistical significance.

## 3. Results

### 3.1. Serum NT-proBNP (BNP) Levels in Normal Control Rats and Diabetes Rats

The serum BNP concentration in the diabetic control group was significantly higher than that in the normal control group (41.07 ± 11.18*vs.*531.33 ± 41.68, *p* < 0.01).

### 3.2. General Phenotypes of Rats, Changes in Body Weight and Blood Glucose, and Blood Lipid Levels

The rats in the diabetic model group were generally in poor condition and bad mental state with slow response, polydipsia, polyuria, weight loss, and cataract compared with those in the control group. Before modeling, the weights of rats in each group increased steadily with no significant difference in their weights between groups. After modeling, the weight of the rats in the model group decreased while the weight in the normal control group increased most heavily, and the weight in the normal administration group was lower than that in the normal control group (*p* < 0.05). As diabetic rats exhibited increased blood glucose levels, early or late administration of dapagliflozin noticeably decreased the levels significantly (*p* < 0.05). There was no significant difference in blood glucose between the normal control group and the normal administration group (*p* > 0.05), but the blood glucose in the early administration group was lower than that in the late administration group (*p* < 0.05). Apart from blood glucose, the model group had elevated blood lipid concentration compared with the normal control group (*p* < 0.05), and the concentration in the normal administration group decreased (*p* < 0.05). The elevated lipid levels in the diabetic rats were decreased by early or late treatment with dapagliflozin (*p* < 0.05), but there was no significant difference between the two model administration groups (*p* > 0.05). See Table 1 and Figure 1.

### 3.3. Electrocardiogram and Its Related Parameters in Rats

As shown in Table 2, the heart rate of rats in the diabetic model group decreased significantly (*p* < 0.05), while the rate was restored in the presence of dapagliflozin and early administration of the drug resulted in greater increase in heart rate (*p* < 0.05). The rats in the diabetic control group had ventricular premature beats and ventricular tachycardia, which were not found in other groups. The QRS wave was widened, and QT interval was prolonged in diabetic control rats (*p* < 0.05). These parameters were shortened in the early administration group and the late administration group, especially early administration group where QRS wave and QT interval declined dramatically compared with in the diabetic control group and the late administration group (*p* < 0.05).

The article "Dapagliflozin Improves Diabetic Cardiomyopathy by Modulating the Akt/mTOR Signaling Pathway" was retracted in 2023. Reasons: unreliable results or conclusions; concerns about the data; concerns about the peer review; concerns about the citations.

### 3.4. HE Staining Results of Myocardial Tissue

The HE results showed that cardiomyocytes in the normal control group were arranged orderly and evenly, myocardial nucleus and cytoplasm were stained clearly, and there was no obvious myocardial fibrosis. There was no significant difference in these characteristics between the normal administration group and the normal control group. In the diabetic control group, myocardial cells were arranged in disorder with increased myocardial interstitial fibers and myocardial cell fibrosis. These disorders were greatly alleviated by early administration of dapagliflozin rather than later administration. In the late administration group, we still found disordered arrangement of cardiomyocytes and obvious cellular edema and fibrosis. See Figure 2.

### 3.5. Cx43 Expression (Immunohistochemical and Western Blot)

Immunohistochemical staining showed that cardiomyocytes were arranged orderly in the normal control group, identifying dense and regular expression of Cx43 mainly in the intercalated disc of myocardium. Dapagliflozin rarely altered these features in the control group with no significant difference between the normal administration group and the normal control group. In the diabetic control group, the myocardial cells were enlarged and disordered, and the expression of Cx43 was dispersed in the cytoplasm of the myocardium. Importantly, early dapagliflozin treatment greatly restored the myocardial cell arrangement and gathered the expression of Cx43 to the irrigation area, which was similar to that in the normal control group. The expression level of Cx43 in myocardial cells of the late administration group was higher than that of the model group, but lower than that of the control group.

There was no significant difference in Cx43 protein expression between the normal control group and the normal administration group (*p* > 0.05). The expression level of Cx43 protein in ventricular myocytes decreased significantly in diabetic rats relative to healthy ones (*p* < 0.05), and the expression was improved significantly by the treatment of dapagliflozin (*p* < 0.05), with higher expression of Cx43 in the early administration group (*p* < 0.05). See Figure 3.

The article "Dapagliflozin Improves Diabetic Cardiomyopathy by Modulating the Akt/mTOR Signaling Pathway" was retracted in 2023. Reasons: unreliable results or conclusions; concerns about the data; concerns about the peer review; concerns about the citations.

### 3.6. mTOR Protein Expression

Injection of dapagliflozin did not cause a significant change in the expression of mTOR in the healthy rats (*p* > 0.05). The mTOR expression was significantly decreased in the diabetic group relative to the normal group (*p* < 0.05). Compared with the diabetic rats, the expression level of mTOR in the early and late administration groups increased significantly (*p* < 0.05) with the higher level in the early administration group (*p* < 0.05). See Figure 4.

### 3.7. p62 Protein Expression

There was no significant difference in protein expression of p62 between the normal control group and the normal administration group (*p* > 0.05), but compared with these two groups, the level of p62 protein in the diabetic control group increased significantly (*p* < 0.05). Moreover, early or late administration of dapagliflozin dramatically decreased the level of p62 protein (*p* < 0.05), with early treatment exhibiting more significantly inhibitory effect (*p* < 0.05). See Figure 5.

### 3.8. Akt Protein Expression

Compared with the normal control group, there was no significant change in the expression of Akt protein in the normal administration group (*p* > 0.05), but the expression level of Akt protein was significantly inhibited in the diabetic control group (*p* < 0.05). Compared with the diabetic control group, the early administration group and the late administration group had higher protein expression of Akt increased significantly (*p* < 0.05). See Figure 6.

### 3.9. LC3-II Protein Expression

As for LC3-II expression, the difference between the normal control group and the normal administration group as well as the control group did not reach significance (*p* > 0.05), but LC3-II protein expression in the diabetic control group was significantly increased (*p* < 0.05). It was found that dapagliflozin treatment resulted in enhancement of LC3-II expression in the diabetic rats (*p* < 0.05), with greater effect in the early administration group (*p* < 0.05). See Figure 7.

## 4. Discussion

The onset of diabetes is hidden and usually presents only metabolic dysfunction in the early stage, including hypertension, insulin resistance, oxidative stress, and autophagy. Many patients develop diabetes after the occurrence of complications [17]. Complications of diabetes include renal failure, retinopathy, neuropathy, and cardiovascular and cerebrovascular diseases. These complications seriously affect the quality of life of the patients. DCM is early manifested by myocardial fibrosis, ventricular stiffness, and cardiac enlargement without obvious clinical symptoms.

The article "Dapagliflozin Improves Diabetic Cardiomyopathy by Modulating the Akt/mTOR Signaling Pathway" was retracted in 2023. Reasons: unreliable results or conclusions; concerns about the data; concerns about the peer review; concerns about the citations.

During diabetes, the patients will undergo structural changes of the heart, cardiac systolic and diastolic dysfunction, and heart failure [18]. The ultrastructure of the diabetic rats (induced by STZ) changed abnormally at 8-12 weeks, and the heart function changed at 6-14 weeks [19]. Therefore, this experiment was only carried out 16 weeks after the establishment of diabetes rat model, and relevant laboratory tests were carried out to better explore the relevant pathological mechanism and pharmacological effects.

In the present study, we assayed that the blood glucose level, water consumption, and urine volume of diabetes rats increased significantly, but their weight decreased significantly. At the end of this experiment, almost all diabetes rats had the symptoms of lethargy and cataract complications, and the blood lipid increased significantly. HE results depicted orderly arrangement of ventricular myocytes in the normal control group and clear staining of myocardial nucleus and cytoplasm without obvious myocardial fibrosis. In the diabetic group, ventricular myocytes were seriously damaged, myocardial cells were disordered and deformed, cell volume and intercellular space increased, and interstitial fibrosis was serious.

Dapagliflozin functions in the body through inhibition of glucose reabsorption and promotion of the excretion of in urine when hindering the high-glucose transporter SGLT2 in the renal proximal tubule [1]. Dapagliflozin has many mechanisms to protect cardiomyocytes such as blood glucose control effects and protective effect on heart failure, cardiovascular mortality [7, 20], and cardiovascular mortality or hospitalization due to heart failure with safety [21]. Dapagliflozin is indicated to significantly improve health conditions related to heart failure, alleviating symptoms and improving physical function and quality of life which lasts for a long time [22].

Dapagliflozin has a variety of mechanisms to protect cardiomyocytes. By inhibiting the oxidative stress mediated by nicotinamide adenine dinucleotide phosphate (NADPH) oxidase, it obviously ameliorated the cardiac dysfunction, improved myocardial fibrosis, apoptosis, and oxidase stress in vivo, and reduced the enhanced level of reactive oxygen species and cell death of H9c2 cells [23]. Besides, the dapagliflozin can improve the biochemical indexes related to cardiac function, including malondialdehyde (MDA), glutathione (GSH), and catalase (CAT), proinflammatory mediators (NF-*κ*B and tumor necrosis factor-*α* (TNF-*α*)), and apoptotic effectors (caspase-3). In addition, it can restore the oxidant/antioxidant balance and attenuates inflammation and downregulates the levels of apoptosis key elements in myocardial tissue [24]. Dapagliflozin obviously improves myocardial hypertrophy caused by T2DM by reducing blood glucose and the expression of calpain-1 in cardiomyocytes [25]. Herein, our experiment was to explore whether dapagliflozin recovered autophagy through the Akt/mTOR signaling pathway and to observe the expression and distribution of Cx43 in ventricular myocytes upon treatment.

The article "Dapagliflozin Improves Diabetic Cardiomyopathy by Modulating the Akt/mTOR Signaling Pathway" was retracted in 2023. Reasons: unreliable results or conclusions; concerns about the data; concerns about the peer review; concerns about the citations.

We found that blood glucose decreased significantly within one week after treatment with dapagliflozin in the early administration group and the late administration group, and weight was well controlled. The blood glucose level in these two groups at the end of the experiment declined dramatically compared with that in the diabetic model group as the early administration group exhibited greater effect. Apart from blood glucose, the lipid levels following dapagliflozin treatment were also significantly reduced.

The proportion of complications in the late administration group was similar to that in the diabetic group. Mild complications occurred in rats in the early administration group, and fewer rats had complications of listlessness and cataracts. Such improvement in the complication is largely attributable to the better control of blood glucose in the early stage of the disease.

HE staining showed damaged ventricular myocytes in the early and late administration groups compared with the normal control group, though the pathological changes of cell arrangement, cell edema, and interstitial fibrosis had been improved. The improvement of myocardial lesions in the early administration group was more significant; Shi's study had similar report [26].

The expression of cardiac Cx is influenced by many factors, such as hypertension, diabetes, myocardial remodeling, and heart failure [27]. Cx is essential for coordinating myocardial excitation and contraction to maintain normal cardiac function [28]. In the present study, immunohistochemistry showed a reduction in the expression of Cx43 in ventricular myocytes of the diabetic group relative to the normal control group, and the lateral of Cx43 in cardiomyocytes could be also observed. Compared with the diabetic control group, the fluorescence of Cx43 in ventricular myocytes obviously increased upon treatment with dapagliflozin. The results by Western blot further confirmed downregulation of Cx43 expression in ventricular myocytes of the diabetic control group compared with the normal control group, and dapagliflozin could improve or reverse Cx43 expression. Interestingly, dapagliflozin rarely affected the expression of Cx43 in ventricular myocytes of normal rats. The results of ECG indicated that the heart rate, QRS wave width, and QT interval were significantly abnormal in the diabetic control group, which were improved by administration of dapagliflozin. The effect of dapagliflozin on ECG-related indexes is consistent with that of dapagliflozin on the regulation of Cx43 in ventricular myocytes.

The article "Dapagliflozin Improves Diabetic Cardiomyopathy by Modulating the Akt/mTOR Signaling Pathway" was retracted in 2023. Reasons: unreliable results or conclusions; concerns about the data; concerns about the peer review; concerns about the citations.

The disorder of Cx43 distribution and abnormal expression are an important pathogenic mechanism to arrhythmia caused by various heart diseases [29]. Cx43 is the main connexin of ventricular myocytes. The lateral Cx43 distribution (remodeling) is a major cause of reduced cardiac conduction reserve and ventricular arrhythmia [30]. Cx43 remodeling is an important pathological mechanism leading to heart failure and arrhythmia [31], and the decrease of Cx43 expression will also increase the incidence of ventricular arrhythmia [32]. Improving the expression and distribution of Cx43 seems to be a new target for the treatment for heart failure and arrhythmia.

The expression and content of Cx43 in cardiomyocytes are closely related to the Akt/mTOR signaling pathway [12]. Autophagy is the main intracellular degradation system and is a process of cell self-degradation and recycling of intracellular components [33]. The amount of LC3-II is closely correlated with the number of autophagosomes, serving as a good indicator of autophagosome formation [34]. Simple comparison of LC3-I and LC3-II, or summation of LC3-I and LC3-II for ratio determinations, may not be appropriate, and rather, the amount of LC3-II can be compared between samples [35]. Measurement of p62 seems an alternative method for detecting the autophagic flux [36].

Therefore, we measured LC3-II in samples in this experiment. Western blot showed that the increase of LC3-II in the myocardium of the diabetes control group was accompanied by the increase of p62, indicating that autophagy of myocardial cells in the diabetic group was inhibited. After dapagliflozin administration, p62 and LC3-II were inhibited in varying degrees in both early and late stages, suggesting that dapagliflozin administration might recover autophagy and alleviate myocardial damage in diabetes rats. The expression of Akt and mTOR decreased in the diabetic group, but in the early and late administration groups, the expression of Akt and mTOR recovered after dapagliflozin administration, suggesting that the regulatory mechanism of dapagliflozin on autophagy may be related to the Akt/mTOR signaling pathway.

The article "Dapagliflozin Improves Diabetic Cardiomyopathy by Modulating the Akt/mTOR Signaling Pathway" was retracted in 2023. Reasons: unreliable results or conclusions; concerns about the data; concerns about the peer review; concerns about the citations.

Upregulation of autophagy can reduce cardiac remodeling and dysfunction in DCM, thus hindering the progression of DCM [37]. The Akt/mTOR signaling pathway plays a regulatory role in autophagy and provides a new therapeutic strategy for many diseases, including diabetes, cancer, and neurodegenerative diseases [38].

## 5. Conclusions

Dapagliflozin may be a specific drug for the prevention and administration of DCM. As a new hypoglycemic agent, dapagliflozin can improve blood lipids and body weight in DCM and has a certain cardioprotective effect. This effect may enhance autophagy through the Akt/mTOR signaling pathway and improve the expression and distribution of Cx43 in ventricular myocytes. However, the safety and efficacy of dapagliflozin in the administration for DCM still need more clinical data for verification, and its potential mechanism needs further exploration.

## Figures and Tables

**Figure 1:** Changes in (a) body weight and (b) blood sugar in rats.

**Figure 2:** HE staining of rat hearts in each group (×400): (a) normal control group, (b) normal administration group, (c) diabetes control group, (d) early administration group, and (e) late administration group.

**Figure 3:** Immunohistochemical staining for Cx43 (×400): A: normal control group, B: normal administration group, C: diabetes control group, D: early administration group, and E: late administration group. ^∗^*p* < 0.05 vs. A; ^&^*p* > 0.05*vs*. A; ^#^*p* < 0.05*vs*. C; ^@^*p* < 0.05*vs*. D.

**Figure 4:** Difference in the expression levels of mTOR proteins: A: normal control group, B: normal administration group, C: diabetes control group, D: early administration group, and E: late administration group. ^∗^*p* < 0.05*vs.* A; ^&^*p* > 0.05*vs.* A; ^#^*p* < 0.05 vs. C; ^@^*p* < 0.05*vs.* D.

**Figure 5:** Relative expression levels of p62 protein in the ventricles of rats in each group: A: normal control group, B: normal administration group, C: diabetes control group, D: early administration group, and E: late administration group. ^∗^*p* < 0.05*vs*. A; ^&^*p* > 0.05*vs*. A; ^#^*p* < 0.05*vs*. C; ^@^*p* < 0.05*vs*. D.

**Figure 6:** Difference in the expression levels of Akt proteins: A: normal control group, B: normal administration group, C: diabetes control group, D: early administration group, and E: late administration group. ^∗^*p* < 0.05*vs.* A; ^&^*p* > 0.05*vs*. A; ^#^*p* < 0.05*vs.* C.

**Figure 7:** Difference in the expression levels of LC3 proteins: A: normal control group, B: normal administration group, C: diabetes control group, D: early administration group, and E: late administration group. ^∗^*p* < 0.05*vs.* A; ^#^*p* < 0.05*vs.* C; ^@^*p* < 0.05*vs.* D.

The article "Dapagliflozin Improves Diabetic Cardiomyopathy by Modulating the Akt/mTOR Signaling Pathway" was retracted in 2023. Reasons: unreliable results or conclusions; concerns about the data; concerns about the peer review; concerns about the citations.

**Table 1:** Weight, blood glucose, and blood lipids of rats at the end of the experiment.

	A (*n* = 10)	B (*n* = 10)	C (*n* = 10)	D (*n* = 10)	E (*n* = 10)
Body weight (g)	443.02 ± 14.97	375.56 ± 10.54^∗^	260.39 ± 23.98^∗^	317.31 ± 14.25^∗^^#^	347.08 ± 13.18^∗^^#^
Blood glucose (mmol/L)	3.84 ± 0.43	4.07 ± 0.43^&^	28.71 ± 2.81^∗^	5.69 ± 0.86^∗^^#^	9.24 ± 1.07^∗^^#@^
TC (mg/dL)	1.34 ± 0.13	1.07 ± 0.10^∗^	6.28 ± 0.77^∗^	4.08 ± 0.26^∗^^#^	4.23 ± 0.19^∗^^#^
TG (mg/dL)	0.84 ± 0.11	0.68 ± 0.04^∗^	2.40 ± 0.26^∗^	1.08 ± 0.18^∗^^#^	1.62 ± 0.18^∗^^#^
LDL-C (mg/dL)	0.28 ± 0.04	0.23 ± 0.04^∗^	1.09 ± 0.16^∗^	0.46 ± 0.07^∗^^#^	0.52 ± 0.09^∗^^#^
HDL-C (mg/dL)	0.91 ± 0.09	0.87 ± 0.09^∗^	1.38 ± 0.19^∗^	0.64 ± 0.08^∗^^#^	0.57 ± 0.08^∗^^#^

A: normal control group; B: normal administration group; C: diabetes control group; D: early administration group; E: late administration group; TC: total cholesterol; TG: triglyceride; HDL-C: high-density lipoprotein; LDL-C: low-density lipoprotein. ^∗^*p* < 0.05*vs.* A; ^#^*p* < 0.05*vs*. C; ^&^*p* > 0.05*vs*. A; ^@^*p* < 0.05*vs*. D.

**Table 2:** Electrocardiogram indexes of rats in each group.

	A (*n* = 10)	B (*n* = 10)	C (*n* = 10)	D (*n* = 10)	E (*n* = 10)
Heart rate (bpm)	381.40 ± 12.14	366.50 ± 6.47	187.88 ± 11.80^∗^	345.75 ± 15.37^∗^^#^	323.11 ± 12.60^∗^^#&^
QRS wave (ms)	36.82 ± 0.13	37.39 ± 0.32	73.53 ± 2.56^∗^	37.17 ± 0.87^#^	40.75 ± 0.33^∗^^#&^
QT interval (ms)	57.29 ± 0.13	58.70 ± 1.04	107.27 ± 5.75^∗^	58.78 ± 0.12^#^	65.45 ± 0.52^∗^^#&^

A: normal control group; B: normal administration group; C: diabetes control group; D: early administration group; E: late administration group. ^∗^*p* < 0.05*vs*. A; ^#^*p* < 0.05*vs*. C; ^&^*p* < 0.05*vs.* D.

## Data Availability

The data used to support the findings of this study are available from the corresponding author upon request.
